The article "The Effects of Physical Exercise on Cognition: How Heart Rate Variability Can Predict Cognitive Performances" was retracted in 2021. Reasons: results that could not be reproduced; errors in the methods.

# The Effects of Physical Exercise on Cognition: How Heart Rate Variability Can Predict Cognitive Performances

**DOI:** 10.3389/fnhum.2020.00312

**Published:** 2020-08-31

**Authors:** Giovanna Sannino, Ivanoe De Falco, Giuseppe De Pietro, Saverio Stranges

**Affiliations:** ^1^ICAR, National Research Council of Italy, Naples, Italy; ^2^Department of Epidemiology and Biostatistics, Schulich School of Medicine and Dentistry, Western University, London, ON, Canada; ^3^Department of Family Medicine, Schulich School of Medicine and Dentistry, Western University, London, ON, Canada; ^4^Department of Population Health, Luxembourg Institute of Health, Strassen, Luxembourg

**Keywords:** cognition, physical exercise, heart rate variability, prediction of cognitive performances, pilot study

## Abstract

**Objectives:** Investigate and identify the relationship between physical exercise and cognitive performance measured by using different cognitive tests taken from Cambridge Brain Science (CBS).

**Methods:** Thirty subjects, divided into two groups (aerobic and effort), undergo twelve cognitive tests from CBS. A comparison between the pre- and post-exercise results in terms of cognitive performance differences is carried out. Regression analysis between Heart Rate Variability (HRV) features and CBS tests results is performed.

**Results:** In most CBS tests, there is an improvement, or at least a confirmation, of the subject's cognitive ability, for both groups. Reasoning (80–100%), concentration (80–87%), and planning tests (93–100%) seem to undergo critical positive changes. The regression analysis, performed by using a set of different algorithms, has demonstrated that it is possible, by monitoring the HRV during the exercise, to predict to some extent the cognitive performance, i.e., the CBS tests results. The best performing regression algorithms are Simple Linear (Quade Test—aerobic group: 2.098, effort group: 3.350, both groups: 2.747) and REPTree (Quade Test—aerobic group: 2.955, effort group: 3.315, both groups: 3.121). The statistical analysis has proved that physical activity is statistically useful for the subjects in improving their cognitive performance.

**Conclusions:** This study has numerically appraised the improvement, the conservation, or the worsening on different aspects of cognition. The found mathematical relationship between physical exercise and cognitive performance suggests that it is possible to predict the beneficial effect of various exercises on executive and attentive control.

## 1. Introduction

The importance of exercise to overall well-being is documented in the scientific literature. Regular exercise is essential for sustaining a healthy body weight and can help in the maintenance of normal blood lipid levels and blood pressure (Fletcher et al., 1992). The benefits of exercise extend beyond physiological changes; exercise is also advantageous to mental health, having been shown to improve self-esteem and self-confidence and to reduce symptoms of depression (Fletcher et al., 1992). The helpfulness of exercise is so systematic and profound that it is recommended in the prevention and management of various medical conditions, including cardiovascular disease, metabolic syndrome, osteoporosis, a number of neoplastic diseases, and various mental illnesses, such as anxiety (Fletcher et al., 1992). However, an often-overlooked aspect of exercise is the effect it has on cognition and the brain.

The article "The Effects of Physical Exercise on Cognition: How Heart Rate Variability Can Predict Cognitive Performances" was retracted in 2021. Reasons: results that could not be reproduced; errors in the methods.

In fact, there is increasing evidence that exercise can have drastic effects on almost all aspects of brain health, including improved learning and memory, reduced symptoms of depression, better outcomes associated with brain injury, and delayed onset and magnitude of cognitive decline associated with various neurodegenerative diseases (Cotman et al., 2007).

Literature shows more and more papers aiming at linking physical activity to improvements in brain function and cognition, as for example (Luft et al., 2009; Paterson and Warburton, 2010; Ahlskog et al., 2011; Erickson et al., 2011; Luque-Casado et al., 2013; Blondell et al., 2014; Scherder et al., 2014; Bherer, 2015; Prakash et al., 2015; Tsunoda et al., 2015; Bauman et al., 2016; Tivadar, 2017). Research carried out on animals shows the positive effect of enriched environments, including access to exercise equipment (such as running wheels) on neuronal growth. The same effect is shown when neural systems involved in learning and memory are considered. This indicates that physically active behaviors have an effect both on the cognitive function and on the related brain structures (Vaynman and Gomez-Pinilla, 2006). Similar results have been found when research is carried out on humans (Booth and Lees, 2006), with recent research in neuroimaging techniques showing that exercise yields apparent modifications both in structure and in the function of the brain.

However, none of the mentioned studies gives the possibility to predict the cognitive performance of the subjects. This possibility is what we investigate in this paper, and represents its novelty.

We present a study aiming to investigate the impact on, and the mathematical relationship between, physical activity and cognitive performances. These latter are measured by using a number of different cognitive tests taken from Cambridge Brain Science, the CBS tests^1^. The study, detailed in section 2, involves thirty subjects, divided into two groups, each with specific physical activity, and twelve cognitive tests.

The article "The Effects of Physical Exercise on Cognition: How Heart Rate Variability Can Predict Cognitive Performances" was retracted in 2021. Reasons: results that could not be reproduced; errors in the methods.

As a result of this study, we have been able to create a brand-new data set linking physical activity and the results of the cognitive tests over time. To the best of our knowledge, this is the first data set of this kind, and no other freely available such data sets exist.

Working on this data set, we have conducted different kinds of analysis in section 3. In detail, as described in section 3.1, we have first evaluated how the physical activity impacts on cognitive activities such as reasoning, work memory, and verbal skills. Or rather, we have numerically appraised, both before and after the physical training, the improvement, the conservation, or the worsening on different aspects of cognition, each of them represented by a CBS test. This evaluation has been made in terms of cognitive performance by defining a suitable numerical Δ*Score*.

Additionally, as detailed in section 3.2, we have analyzed if a mathematical relationship exists between physical exercise and cognitive performance. This has been done by studying if a regression model can be found that is able to predict the cognitive performance, i.e., the CBS test scores, by using the Heart Rate Variability (HRV) features monitored during the physical exercise. To perform regression, several algorithms are considered, and the best six, in terms of three different regression quality indexes, are reported.

We have chosen to use the HRV, a non-invasive parameter, because this allows measuring the dynamic autonomic responses during exercise through the analysis of the ElectroCardiogram (ECG) signal, i.e., the HRV, as demonstrated in important studies in the scientific literature (Makivić et al., 2013; Ngandu et al., 2015). These results indicate that it is possible to use the HRV parameters for the analysis of the stress experienced by the body during the training phase, and for better understanding the physiological recovery following the training. As a matter of fact, it is sensible to hypothesize that modifications in the Autonomic Nervous System (ANS) patterns, represented by modifications in the HRV, might act as helpful parameters for the management of both physical fatigue and exercise intensity.

The purpose of finding a mathematical relationship between HRV and cognitive performance is to predict the beneficial effect of various exercise programs (aerobics or muscle strength) on executive and attentive control (work memory, distributed focus, inhibition of response, interference on control).

This is a particularly relevant research activity aiming to demonstrate if a direct correlation between the trend of HRV and cognitive performance exists. In fact, if demonstrated, it would be possible to design prevention activities based on personalized exercise programs that, using HRV analysis, are optimized for the improvement of cognitive abilities.

The article "The Effects of Physical Exercise on Cognition: How Heart Rate Variability Can Predict Cognitive Performances" was retracted in 2021. Reasons: results that could not be reproduced; errors in the methods.

Finally, as mentioned in section 3.3, a statistical analysis is run to: (i) understand if the physical activity is statistically useful for the subjects in improving their performance at solving the 12 CBS tests; and (ii) to evaluate the quality of the regression models.

## 2. Methods

### 2.1. Ethics Statement

This study has been conducted in compliance with the World Medical Association Declaration of Helsinki on Ethical Principles for Medical Research Involving Human Subjects (World Medical Association, 2008).

The protocol guidelines of the study have been written in conformity with the SPIRIT 2013 Statement (Chan et al., 2013), and, before the start of the experimental session, the participants read and signed an informed consent statement. Suitable information was given to them about their right to quit the experiment whenever they wanted, and each of the subjects was informed in a detailed way about the goal of this study when the experimental session ended. Finally, all the data from all the participants were examined, filed, and described in a completely anonymous form.

### 2.2. The Recruitment: Participants and Procedure for the Data Acquisition

We recruited 30 healthy participants (age range: 18–48 years old), of which 18 males and 12 females.

In order to be considered suitable for the trial process, the subjects had to comply with these criteria:

- Adults aged over 18 years;
- Subjects with no level of physical fitness as defined in the normative values of the American College of Sports Medicine (Sharp, 1993);
- Subjects being no professional athletes;
- No people suffering from any pathological cardiovascular conditions, neurological or psychiatric disorders or other severe diseases.

The procedure of the study has been outlined in Figure 1.

**Figure 1:** Schema of the protocol performed for the data collection phase.

In the following, we report a brief summary of the phases of the protocol performed for data collection:

**Day 1 :**

- The participant is informed about the purposes of the study and how it will be conducted. Information material is provided, and the participant is invited to sign the informed consent.
- The participant is apprised of the use of the wearable device that she/he should wear during physical activity for the continuous acquisition of the Heart Rate (HR) data, the Zephyr BioHarness BH3 (Zephyr Technology, 2016). Together with the device, detailed instructions are given on how to place the sensor and on how to use it.
- The participant is informed about the 12 cognitive tests of the CBS that they will have to perform after each physical exercise, and about the modality for the on-line compilation through the platform on CBS site^2^.
  Figure 2 shows the 12 cognitive tests used: the green ones are related to the Short Term Memory (STM) cognition, those relating to the reasoning abilities are shown in blue, those relating to verbal skills in red, whereas the purple ones make reference to memory.
- The participant is informed about the scheduling of the activities, which is set as follows:
  **Task 1** - Initial cognitive assessment: day 1;
  **Task 2** - 1st battery of 12 cognitive tests: day 5;
  **Task 3** - 2nd battery of 12 cognitive tests: day 10;
  **Task 4** - 3rd battery of 12 cognitive tests: day 15;
  **Task 5** - 4th battery of 12 cognitive tests: day 20;
  **Task 6** - 5th battery of 12 cognitive tests: day 25;
  **Task 7** - Final cognitive assessment: day 30.
  Between one task and another, the participant is invited to perform a minimum of 3 h of physical exercise (even non-continuative), preferably 1 h per day for 3 days. The type of physical exercise to be performed will depend on the target group to which it will be assigned, which can be either aerobic or effort. If assigned to the aerobic group, the subject must perform a type of aerobic exercise, such as running or cycling. If, instead, the subject is assigned to the effort group, she/he must perform a type of exercise that is short but intense, such as lifting weights, bending, or lifting at the bar. Of the 30 people recruited, 15 were chosen in a random way and allocated to the effort group (Group 1), while the other 15 to the aerobic group (Group 2).
- The initial cognitive assessment is requested on site.

The article "The Effects of Physical Exercise on Cognition: How Heart Rate Variability Can Predict Cognitive Performances" was retracted in 2021. Reasons: results that could not be reproduced; errors in the methods.

**Days 5, 10, 15, 20, and 25 :**

- The participant is asked to send the HR data acquired until now;
- The results of each battery of 12 cognitive tests
  in each day are collected through the CBS platform.

**Day 30 :**

- The participant is asked to send the HR data acquired so far;
- The final cognitive assessment is requested on site;
- The participant will return the instrumentation received.

**Figure 2:** The 12 tests included in the CBS battery: the green ones are related to the Short Term Memory (STM) cognition, those relating to the reasoning abilities are shown in blue, those relating to verbal skills in red, whereas the purple ones make reference to memory. **(A)** Spatial span test. **(B)** Token search test. **(C)** Monkey ladder test. **(D)** Paired associates test. **(E)** Spatial planning test. **(F)** Spatial rotations test. **(G)** Feature match test. **(H)** Interlocking polygons test. **(I)** Odd one out test. **(J)** Digit span test. **(K)** Grammatical reasoning test. **(L)** Double trouble test. All the images in this figure are taken from: https://www.cambridgebrainsciences.com.

### 2.3. The Cognitive Measurements

The current study uses CBS tests^3^ to assess cognitive performance. CBS is a set of 12 on-line tests used to measure different aspects of cognitive function. This collection of tests assesses aspects of inhibition, selective attention, reasoning, verbal STM, spatial working memory, planning, and cognitive flexibility. Together, these tests collectively and comprehensively assess three cognitive domains: STM, reasoning, and verbal abilities, based on behavioral data (from over 44,000 individuals) and neuroimaging studies that have demonstrated that each domain is supported by a separate brain network (Hampshire et al., 2012). They have been validated in patients (Owen et al., 1990, 1991, 1993) and healthy populations (Owen et al., 1996a,b) and have been shown to be sensitive to subtle cognitive changes due to neurodegeneration (Owen et al., 1992, 1993) or pharmacological intervention (Lange et al., 1992; Mehta et al., 2000). In addition, the tests are designed to be engaging to maximize participant compliance. Completion of the battery requires between 35 and 45 min, which is faster and more convenient than many other pen-and-paper neuropsychological batteries. Taken together, the CBS battery is ideal to use in the current study because it is easy and fast to complete, can be used to assess even the most subtle changes in cognition, and the categorization of tests into latent cognitive domains will help to provide an objective definition of exactly which cognitive processes are influenced by physical activity.

Below we give the summary of the CBS tests used in this study, and the cognitive area they are related to.

- **Memory**: Monkey Ladder, Spatial Span, Paired Associates, Digit Span;
- **Reasoning**: Odd One Out, Double Trouble, Grammatical Reasoning;
- **Concentration**: Spatial Rotation, Feature Match, Interlocking Polygons;
- **Planning**: Spatial Planning, Token Search.

### 2.4. The HRV Measurements

The HRV measurements have been extracted from the HR data monitored by using the Zephyr BioHarness BH3 Sensor (Zephyr Technology, 2016). This HR sensor can be used at the gym, on a run, while exercising at home, or during physical therapy. It is small, wearable, and compatible with many Bluetooth devices, and very suitable for personal and clinical use.

All HR data were processed using a Matlab-based software, named Kubios (Tarvainen et al., 2014), designed at the University of Kuopio, Finland. This is a state-of-the-art tool for the extraction and the analysis of the HRV characteristics from the HR data. Through Kubios, a set of parameters was extracted in the Time domain, in the Frequency domain, and in the Non-Linear domain.

The article "The Effects of Physical Exercise on Cognition: How Heart Rate Variability Can Predict Cognitive Performances" was retracted in 2021. Reasons: results that could not be reproduced; errors in the methods.

Before extracting the HRV parameters, each record is cleaned from power line interferences, muscle and movement artifacts, through the use of a cubic spline interpolation procedure (Daskalov and Christov, 1997; Mateo and Laguna, 2000).

The RR- interval, also called the NN-interval, is determined by the distance between two successive heartbeats in a normal rhythm of the ECG signal. As interference may take place between artifacts in the RR interval time series and the analysis of these signals, we decided to use the Kubios Artifacts removal RR filter set to a maximum threshold of 5%.

After filtering, the analysis of the signals took place. In detail, 34 characteristic parameters were extracted, summarized in Table 1.

**Table 1:** HRV features: the features from 1 to 9 are related to the Time domain, the features from 10 to 22 refer to the Frequency domain, while those from 24 to 34 are related to the non-linear domain.

	**Measure**	**Unit**	**Description**
1	MeanRR	ms	The mean of RR intervals
2	STDRR	ms	Standard deviation of RR (NN) intervals
3	MeanHR	1/min	The mean of HRs values
4	STDHR	1/min	Standard deviation of HRs values
5	RMSSD	ms	Square root of the mean squared differences between successive RR intervals
6	NN50	count	Number of successive RR interval pairs that differ more than 50m
7	pNN50	%	NN50 divided by the total number of RR intervals
8	RRtri		The integral of the RR interval histogram divided by the height of the histogram
9	TINN	Ms	Baseline width of the RR interval histogram
10	PeakVLF	Hz	Peak frequencies of the very-low-frequency band
11	PeakLF	Hz	Peak frequency of the Low Frequency (LF) band (0.04–0.15 Hz)
12	PeakHF	Hz	Peak frequency of the High Frequency (HF) band (0.15–0.4 Hz)
13	VLF	ms^2^	Absolute power of the very-low-frequency band (0.0033–0.04 Hz)
14	LF	ms^2^	Absolute powers of LF band, calculated with AR
15	HF	ms^2^	Absolute powers of HF band, calculated with AR
16	Relative VLF	%	Relative power of the very-low-frequency band
17	Relative LF	%	Relative power of the low-frequency band
18	Relative HF	%	Relative power of the high-frequency band
19	Norm. Power LF	nu	Relative power of the low-frequency band in normal units
20	Norm. Power HF	nu	Relative power of the high-frequency band in normal units
21	Total Power	ms^2^	Sum of the energy in the VLF, LF, and HF bands
22	LF/HF	%	Ratio between LF and HF band powers
23	SD1	ms	St. dev. of the Poincarè plot perpendicular to the line of identity
24	SD2	ms	St. dev. of the Poincarè plot along to the line of identity
25	ApEn		Approximate entropy
26	SampEn		Sample entropy
27	D2		Correlation Dimension
28	DFA1		Short-term fluctuation slope in Detrended Fluctuation Analysis
29	DFA2		Long-term fluctuation slope in Detrended Fluctuation Analysis
30	RPLmean	beats	Recurrent Plot (RP) mean line length
31	RPLmax	beats	RP maximum line length
32	RPREC	%	RP Recurrence Rate
33	RPDET	%	RP Determinism
34	RPShan		RP Shannon Entropy

The features from 1 to 9 are related to the Time domain, the features from 10 to 22 refer to the Frequency domain, while those from 24 to 34 are related to the Non-Linear domain.

The article "The Effects of Physical Exercise on Cognition: How Heart Rate Variability Can Predict Cognitive Performances" was retracted in 2021. Reasons: results that could not be reproduced; errors in the methods.

These characteristics were extracted from each HR data acquisition related to each run linked to a single exercise session of each participant.

### 2.5. The Database

The average values of the HRV parameters relative to the runs between two successive batteries of 12 CBS tests have been correlated with the CBS tests results of the second of these batteries.

In practice, referring to Figure 1, for each individual exercise session (Run), a vector of 34 HRV features has been extracted. The average of the HRV characteristics relative to the runs between two successive batteries of 12 CBS tests is then computed.

To better understand the construction mechanism of each database item, let us suppose that the subject performed three exercise runs between day 1, in which she/he underwent the initial cognitive assessment, and day 5, when she/he engages in the first battery of CBS tests. From each HR signal monitored in each of the three exercise runs, 34 HRV features are extracted. So, for each HRV feature, we have three values, one for each exercise run. We have computed the average of these three values. The vector containing the averages of all the HRV features is then put in correlation with the scores of the CBS tests made on Day 5.

Following this procedure, for each subject, we have obtained a number of six items. Each of these latter is constituted as below:

(1) $$\begin{array}{r} item=id;avg(\vec{f\left(HRV\right)}{|}_{1}^{34});\vec{f\left(CBS\right)}{|}_{1}^{12} \end{array}$$

where:

- *id*: is a value from 1 to 30 that unequivocally and anonymously identifies each participant;
- $avg(\vec{f\left(HRV\right)}{|}_{1}^{34})$: is a vector containing the average values of the 34 HRV features computed over the runs performed within two successive batteries of 12 CBS tests;
- $\vec{f\left(CBS\right)}{|}_{1}^{12}$: is the vector containing the CBS test results;

As a result of all the pre-processing phases and of the procedure faced, the data set used in this study consists of 180 items (6 items for 30 subjects), 90 of which related to group 1 (effort group), and 90 to group 2 (aerobic group).

The article "The Effects of Physical Exercise on Cognition: How Heart Rate Variability Can Predict Cognitive Performances" was retracted in 2021. Reasons: results that could not be reproduced; errors in the methods.

## 3. Results

### 3.1. Impact of Physical Exercise on Cognitive Performance

We have performed an analysis to determine whether the different exercise regimes (aerobic vs. effort exercise) had differential effects on cognition, and how they reflected in the change in performance over time. To this aim, for each subject, for the generic i-th CBS test (among the 12) we have defined:

(2) $$\begin{array}{r} \Delta Score_{i}\%=\frac{CBS_{i}\left(day=30\right)-CBS_{i}\left(day=1\right)}{max{\left(CBS\right)}_{i}-min{\left(CBS\right)}_{i}}*100.0{|}_{i=1}^{12} \end{array}$$

where

- *max*(*CBS*)_*i*_: is the maximum among the values obtained by all the subjects over the i-th CBS test;
- *min*(*CBS*)_*i*_: is the minimum among the values obtained by all the subjects over the i-th CBS test.

As shown in Figure 3, we can see that in some cases there has been an improvement in cognitive performance, whereas in others this is not the case. This improvement is different between the two groups, effort and aerobic.

**Figure 3:** Upper pane: Δ*Scores* of each subject belonging to the Group 1 (Effort group) calculated for the 12 CBS tests. Lower pane: Δ*Scores* of each subject belonging to the Group 2 (Aerobic group) calculated for the 12 CBS tests.

To better understand how many subjects have achieved an improvement in cognition from the physical exercise, we report in Table 2 these numerical results expressed in percentage. The most significant percentages are reported in bold. As we can see, tests related to the reasoning, in particular Double Trouble and Grammatical Reasoning, have obtained a significant improvement. In fact, for the Double Trouble all the subjects of group 1 (100%) have achieved better performance at the end of the study (day = 30) with respect to the assessment made at the beginning of the study (day = 1). Meanwhile, for the Grammatical Reasoning, the number of cases in which an improvement has been registered is greater in Group 2 (aerobic), with respect to Group 1 (effort). Good improvements have also been registered for the concentration, especially in the Spatial Rotation test, in which, for both groups, we have an improvement in at least 80% of the subjects. Finally, also for the planning there is a significant improvement in almost all subjects of both groups, in detail in 100% of the subjects for Group 1 (effort) and in 93% of the subjects for Group 2 (aerobic). No important consequences have been registered for the tests related to the memory in both groups. This means that physical exercise does not impact so much on memory performance.

The article "The Effects of Physical Exercise on Cognition: How Heart Rate Variability Can Predict Cognitive Performances" was retracted in 2021. Reasons: results that could not be reproduced; errors in the methods.

**Table 2:** Percentages of subjects who have achieved an improvement, a conservation, or a worsening on the CBS tests results.

	**Group 1**			**Group 2**		

	**Δ > 0**	**Δ = 0**	**Δ < 0**	**Δ > 0**	**Δ = 0**	**Δ < 0**
Digit span	27%	53%	20%	47%	13%	40%
Monkey ladder	33%	27%	40%	33%	33%	33%
Paired association	27%	20%	53%	13%	40%	47%
Spatial span	47%	20%	33%	53%	13%	33%
Double trouble	**100%**	0%	0%	**93%**	7%	0%
Gram. reasoning	60%	7%	33%	**80%**	0%	20%
Odd one out	60%	7%	33%	47%	13%	40%
Features match	**80%**	0%	20%	67%	0%	33%
Interlocking polygons	67%	0%	33%	67%	0%	33%
Spatial rotation	**87%**	0%	13%	**80%**	0%	20%
Token search	47%	0%	53%	47%	20%	33%
Spatial planning	**100%**	0%	0%	**93%**	7%	0%

*Δ Refers to the Δ Score defined in Equation (2)*.

*The most significant percentages are reported in bold*.

### 3.2. The Regression Analysis to Predict the Cognitive Performance

From a hardware viewpoint, all the experiments reported in this paper have been effected on an iMac with High Sierra (Mac OsX 10.13.2) operating system, a 3.6-GHz Intel Core i7 processor, 8GB DDR4 at 2,400 MHz, and a 1 TB hard disk.

We have performed our experiments in the Waikato Environment for Knowledge Analysis (WEKA), version 3.8.1 (Garner, 1995). In it, we have taken advantage of a wide set of regression models coming from artificial intelligence, some already contained in the basic WEKA version, and some others freely downloadable from its repository. We have executed a good number of such models, and we have chosen to report here the best-performing algorithms, i.e., the ones which have achieved the best numerical results in our experiments. These have resulted in being the Support Vector Machine (SVM) (Zeng et al., 2008; Bouguila and Amayri, 2009), the Multi-Layer Perceptron (MLP) Artificial Neural Network (Rumelhart et al., 1988), the Instance-Based K-nearest neighbors (IBk) (Aha et al., 1991), the Reduced Error Pruning Tree (REPTree) (Breslow and Aha, 1997), the Simple Linear and the Additive regression (Stone, 1985).

We have run all the regression models over the data set by performing five-fold cross-validation. This protects us from the overfitting problem by dividing the data set into five folds and estimating regression quality on each fold.

It is important to underline here that we chose not to carry out any parameter tuning phase that could assist us in finding the most appropriate values for the parameters of the different regression algorithms. Also, we chose not to rely on Principal Component Analysis, rather we have made use for the regression of all the 34 HRV features extracted from the signals.

The article "The Effects of Physical Exercise on Cognition: How Heart Rate Variability Can Predict Cognitive Performances" was retracted in 2021. Reasons: results that could not be reproduced; errors in the methods.

Considering that the two types of physical activity impact differently on the same characteristics of HRV, the analysis has been separately performed for each group. Therefore, 12 regression models were identified, each one to predict a single CBS test result for the effort group (Group 1), and other 12 regression models were identified for the aerobic group (Group 2).

To evaluate the regression models used in this study, we have chosen three quality indicators, the Pearson correlation coefficient (ρ), the Mean Absolute Error (MAE), and the Root Mean Square Error (RMSE).

Correlation is a bivariate analysis measuring the strength of association between two variables as well as the direction of this relationship. Given a pair of random variables *y* and ŷ, where *y*_*i*_ is the actual output and ŷ_*i*_ is the model's prediction, ρ is defined as:

(3) $$\begin{array}{r} \rho_{y,ŷ}=\frac{cov\left(y,ŷ\right)}{\sigma_{y}\sigma_{ŷ}} \end{array}$$

where:

- *cov*: is the covariance between *y* and ŷ;
- σ_*y*_: is the standard deviation of *y*;
- σ_ŷ_: is the standard deviation of ŷ

As concerns the strength of the relationship, the value of ρ ranges within −1 and +1, and the higher the value, the better the model. When the value of ρ lies around ±1, a perfect degree of association, be it direct or inverse, is said to exist between the two variables.

In MAE, the error is computed as the average of the absolute differences between the target values and the corresponding predictions. Mathematically, it is calculated using the formula:

(4) $$\begin{array}{r} MAE=\left(1/n\right)\overset{n}{\underset{i=1}{\sum }}|y_{i}-{ŷ}_{i}| \end{array}$$

It is a linear score, so all the individual differences are assigned equal weights. As an example, the difference between 30 and 20 is considered as twice that between 30 and 25.

The RMSE is defined by the equation:

(5) $$\begin{array}{r} RMSE=\sqrt{\left(1/n\right)\cdot \overset{n}{\underset{i=1}{\sum }}{\left(y_{i}-{ŷ}_{i}\right)}^{2}} \end{array}$$

The lower are the values for MAE and RMSE, the better the model is.

As said above, among all the models tested, we report the results achieved by the best six models, namely SVM, MLP, REPTree, IBk, Simple Linear, and Additive Regression. The numerical results, obtained over the train and test sets, are shown in the tables from Tables 3–5 in terms of ρ, MAE, and RMSE specified in the equations above. In each of these tables, we show in bold the best values achieved over each CBS test for both train and test sets.

**Table 3:** Numerical results, obtained over train and test sets, related to ρ.

**Group 1**												

	**SVM**		**MLP**		**REPTree**		**IBk**		**Simple linear**		**Additive**	
	**Train**	**Test**	**Train**	**Test**	**Train**	**Test**	**Train**	**Test**	**Train**	**Test**	**Train**	**Test**
Digit span	0.822	−0.368	0.957	0.025	0.805	0.323	0.979	0.121	0.445	**0.370**	**1.000**	−0.251
Monkey ladder	0.772	0.672	**1.000**	0.593	0.917	0.449	0.956	0.632	0.445	**0.730**	0.998	0.225
Paired associates	0.756	**0.514**	0.937	−0.205	0.000	0.000	0.953	−0.267	0.533	0.169	**0.961**	−0.119
Spatial span	0.627	−0.115	0.955	−0.127	0.955	−0.127	**1.000**	−0.292	0.307	−0.249	**1.000**	**0.135**
Double trouble	0.810	0.275	**1.000**	0.239	0.000	0.000	0.986	−0.533	0.403	0.760	**1.000**	**0.774**
Grammatical reasoning	0.734	0.632	**1.000**	0.517	0.509	0.290	**1.000**	0.223	0.520	**0.856**	0.975	0.292
Odd one out	0.869	0.346	**1.000**	−0.123	0.000	0.000	0.966	0.127	0.459	**0.538**	**1.000**	0.174
Feature match	0.800	0.304	**1.000**	0.007	0.503	0.517	**1.000**	**0.701**	0.466	0.535	0.994	0.493
Interlocking polygons	0.885	0.003	0.969	−0.085	0.738	−0.419	**1.000**	−0.276	0.501	0.042	**1.000**	**0.102**
Spatial planning	0.627	−0.115	0.955	−0.127	0.000	0.000	**1.000**	−0.292	0.307	−0.249	**1.000**	**0.135**
Token search	0.686	−0.098	**1.000**	0.131	0.000	0.000	**1.000**	−0.042	0.486	**0.166**	0.961	0.092
Spatial rotations	0.759	−0.080	0.984	0.045	0.000	0.000	0.975	**0.222**	0.410	−0.717	**1.000**	−0.749
**Group 2**												
	**Train**	**Test**	**Train**	**Test**	**Train**	**Test**	**Train**	**Test**	**Train**	**Test**	**Train**	**Test**
Digit span	0.743	−0.114	0.969	−0.118	0.000	0.000	**1.000**	−0.123	0.540	**0.225**	**1.000**	−0.151
Monkey ladder	0.736	0.263	0.996	0.299	0.000	0.000	**1.000**	**0.404**	0.372	0.063	0.932	−0.325
Paired associates	0.286	0.070	0.971	0.511	0.000	0.000	0.969	**0.597**	0.230	0.493	**1.000**	0.392
Spatial span	0.746	0.047	**1.000**	0.256	0.576	0.092	**1.000**	−0.121	0.473	**0.144**	0.915	0.009
Double trouble	0.749	0.151	0.974	0.460	0.000	0.000	**1.000**	**0.727**	0.532	0.126	0.966	0.095
Grammatical reasoning	0.651	−0.111	0.990	**0.276**	0.850	0.147	**0.992**	0.188	0.390	0.090	0.991	−0.170
Odd one out	0.791	−0.373	0.949	−0.197	0.000	0.000	**0.987**	−0.279	0.490	−0.302	0.971	**0.010**
Feature match	0.601	**0.607**	**1.000**	0.204	0.000	0.000	0.979	0.296	0.314	0.179	0.982	−0.258
Interlocking polygons	0.704	0.093	**1.000**	0.044	0.648	0.054	**1.000**	**0.343**	0.378	−0.137	0.938	0.103
Spatial planning	0.746	0.047	**1.000**	−0.256	0.576	0.092	**1.000**	−0.121	0.473	**0.144**	0.915	0.009
Token search	0.736	**0.397**	**1.000**	−0.425	0.000	0.000	0.985	0.145	0.298	−0.131	0.961	0.354
Spatial rotations	0.780	**0.024**	0.987	−0.110	0.485	−0.382	**1.000**	−0.076	0.390	−0.345	0.954	−0.079

*The values in bold are the best values achieved over each CBS test for both train and test sets*.

The article "The Effects of Physical Exercise on Cognition: How Heart Rate Variability Can Predict Cognitive Performances" was retracted in 2021. Reasons: results that could not be reproduced; errors in the methods.

**Table 4:** Numerical results, obtained over train and test sets, related to MAE.

**Group 1**												

	**SVM**		**MLP**		**REPTree**		**IBk**		**Simple linear**		**Additive**	
	**Train**	**Test**	**Train**	**Test**	**Train**	**Test**	**Train**	**Test**	**Train**	**Test**	**Train**	**Test**
Digit span	0.482	1.763	0.158	1.865	0.828	1.310	**0.000**	1.564	1.228	**1.257**	0.162	1.553
Monkey ladder	0.355	0.407	0.005	0.645	0.260	0.576	**0.000**	0.446	0.611	**0.346**	0.019	0.938
Paired associates	0.387	**0.595**	0.243	0.932	0.716	0.669	**0.000**	1.199	0.635	0.784	0.071	1.053
Spatial span	0.511	0.772	0.016	0.842	0.016	0.842	**0.000**	1.002	0.770	**0.766**	0.102	1.120
Double trouble	6.212	14.371	3.939	18.727	14.379	9.334	**0.000**	14.583	14.013	**7.378**	2.250	7.845
Grammatical reasoning	2.062	4.065	0.065	5.734	3.055	5.630	**0.000**	6.340	4.227	**3.446**	0.471	6.346
Odd one out	1.159	3.163	0.031	5.037	3.158	2.802	**0.000**	3.961	2.530	**2.603**	0.447	3.299
Feature match	12.623	40.143	0.851	61.627	21.039	**32.286**	**0.000**	37.289	22.212	41.637	3.716	40.893
Interlocking polygons	5.118	83.118	0.714	41.409	12.719	26.773	**0.000**	30.596	16.250	26.687	3.146	**18.189**
Spatial planning	0.511	0.772	0.016	0.842	0.808	**0.633**	**0.000**	1.002	0.770	0.766	0.102	1.120
Token search	0.601	1.879	0.007	1.899	1.193	**1.550**	**0.000**	1.682	1.041	1.767	0.196	1.952
Spatial rotations	13.929	54.789	10.577	86.243	27.419	**30.149**	**0.000**	40.039	25.341	37.351	3.796	48.654
**Group 2**												
	**Train**	**Test**	**Train**	**Test**	**Train**	**Test**	**Train**	**Test**	**Train**	**Test**	**Train**	**Test**
Digit span	1.634	1.546	1.215	3.919	2.740	**1.214**	**0.000**	3.628	3.773	4.629	0.422	1.374
Monkey ladder	0.603	1.050	0.391	1.516	1.195	0.825	**0.000**	**0.716**	1.152	0.851	0.362	1.389
Paired associates	2.644	**1.225**	0.969	4.178	4.027	2.416	**0.000**	5.004	4.581	2.130	1.791	3.874
Spatial span	0.357	2.593	0.028	3.046	0.652	2.478	**0.000**	2.466	0.751	**2.372**	0.240	2.466
Double trouble	8.474	13.615	2.016	12.041	15.649	10.008	**0.000**	**8.619**	17.038	16.447	3.580	16.928
Grammatical reasoning	2.238	6.686	0.729	6.252	1.611	5.685	**0.000**	6.072	3.520	**5.613**	1.087	7.155
Odd one out	1.061	3.401	0.217	4.667	2.308	**2.692**	**0.000**	3.867	1.882	3.502	0.831	3.003
Feature match	19.040	**35.524**	8.971	48.518	30.590	43.423	**0.000**	49.285	27.443	41.263	11.028	47.818
Interlocking polygons	11.691	25.903	2.695	34.370	17.917	**20.002**	**0.000**	26.527	22.335	20.916	7.757	23.353
Spatial planning	0.357	2.593	0.028	3.046	0.652	2.478	**0.000**	2.466	0.751	**2.372**	0.240	2.466
Token search	0.956	2.015	0.046	3.653	2.043	2.002	**0.000**	2.167	1.859	2.156	0.587	**1.927**
Spatial rotations	11.381	39.601	5.561	57.657	21.031	42.366	**0.000**	46.959	22.505	**39.065**	6.985	45.483

*The values in bold are the best values achieved over each CBS test for both train and test sets*.

The article "The Effects of Physical Exercise on Cognition: How Heart Rate Variability Can Predict Cognitive Performances" was retracted in 2021. Reasons: results that could not be reproduced; errors in the methods.

**Table 5:** Numerical results, obtained over train and test sets, related to RMSE.

**Group 1**												

	**SVM**		**MLP**		**REPTree**		**IBk**		**Simple linear**		**Additive**	
	**Train**	**Test**	**Train**	**Test**	**Train**	**Test**	**Train**	**Test**	**Train**	**Test**	**Train**	**Test**
Digit span	0.941	2.338	0.261	2.606	0.958	1.735	**0.000**	1.931	1.470	**1.607**	0.181	2.286
Monkey ladder	0.654	0.495	0.006	0.832	0.382	0.761	**0.000**	0.707	0.806	**0.451**	0.032	1.104
Paired associates	0.593	**0.715**	0.368	1.098	0.865	0.813	**0.000**	1.255	0.697	0.870	0.092	1.288
Spatial span	0.832	0.990	0.021	1.034	0.021	1.034	**0.000**	1.207	0.978	**0.866**	0.128	1.276
Double trouble	12.012	20.763	4.733	22.474	17.863	13.182	**0.000**	19.834	17.862	**8.246**	2.857	10.060
Grammatical reasoning	4.225	5.078	0.087	7.165	5.477	6.707	**0.000**	7.281	5.372	**4.099**	0.675	6.662
Odd one out	2.054	3.988	0.036	8.136	3.789	3.291	**0.000**	4.758	3.491	**3.094**	0.647	4.446
Feature match	19.885	50.603	1.106	77.792	26.870	44.509	**0.000**	**43.991**	27.603	49.953	4.563	45.344
Interlocking polygons	9.910	117.538	1.020	51.443	16.021	32.376	**0.000**	34.413	19.685	33.091	3.855	**23.408**
Spatial planning	0.832	0.990	0.021	1.034	1.021	**0.725**	**0.000**	1.207	0.978	0.866	0.128	1.276
Token search	0.981	2.509	0.008	2.549	1.373	**1.990**	**0.000**	2.614	1.170	2.141	0.271	2.660
Spatial rotations	24.112	62.291	13.223	143.750	33.254	**39.048**	**0.000**	44.948	30.968	43.005	5.050	61.226
**Group 2**												
	**Train**	**Test**	**Train**	**Test**	**Train**	**Test**	**Train**	**Test**	**Train**	**Test**	**Train**	**Test**
Digit span	6.552	1.972	1.621	8.720	8.089	1.584	**0.000**	10.258	6.301	5.747	0.487	**1.575**
Monkey ladder	1.052	1.328	0.442	1.694	1.554	**1.083**	**0.000**	1.084	1.382	1.176	0.442	1.949
Paired associates	12.204	**1.619**	1.130	7.344	11.864	2.637	**0.000**	15.536	11.452	2.898	3.533	11.200
Spatial span	0.762	6.741	0.036	7.459	0.859	6.701	**0.000**	7.351	0.884	**6.536**	0.293	6.729
Double trouble	18.144	17.186	2.429	16.340	26.201	14.090	**0.000**	**10.211**	23.233	18.370	4.566	20.857
Grammatical reasoning	3.602	7.882	0.908	7.210	2.463	7.783	**0.000**	7.636	4.337	**6.471**	1.537	9.261
Odd one out	1.729	4.983	0.271	6.335	2.874	**3.788**	**0.000**	5.226	2.647	4.998	0.998	3.955
Feature match	32.704	**61.152**	9.573	73.175	42.161	74.114	**0.000**	69.340	36.938	74.673	13.444	77.258
Interlocking polygons	22.678	29.579	4.139	44.320	24.852	27.111	**0.000**	34.783	31.378	**24.697**	11.072	30.006
Spatial planning	0.762	6.741	0.036	7.459	0.859	6.701	**0.000**	7.351	0.884	**6.536**	0.293	6.729
Token search	1.656	2.477	0.056	4.343	2.287	**2.465**	**0.000**	3.119	2.154	2.709	0.761	2.721
Spatial rotations	19.415	**49.498**	6.757	68.515	27.172	56.026	**0.000**	59.338	27.218	53.906	8.882	52.809

*The values in bold are the best values achieved over each CBS test for both train and test sets*.

The article "The Effects of Physical Exercise on Cognition: How Heart Rate Variability Can Predict Cognitive Performances" was retracted in 2021. Reasons: results that could not be reproduced; errors in the methods.

Over the train set, IBk is, without doubt, the best algorithm. As a matter of fact, for MAE and RMSE it achieves perfect regression, with no error. Also for ρ it often reaches the highest possible final value, i.e., 1.0. On the other hand, the outcomes achieved over the test set present a totally different scenario. This difference in IBk results for the two sets proves that this algorithm is highly afflicted by overfitting. This term is used to express that the IBk regression model achieved is customized to the train set elements, so it faces problems when it has to deal with the never-before-seen test set instances.

### 3.3. Statistical Analysis

Two important issues arise from the results shown above.

The first issue takes into account the results from a cognitive viewpoint. Namely, it raises questions about the usefulness of the physical activity: has this latter statistically helped those subjects improve their performance at solving the 12 tests? If the answer is positive, which kind of activity, effort or aerobic, has been more helpful? And, is it the same for all the tests?

The second issue, instead, concerns the quality of the regression results obtained. Namely, from a statistical viewpoint, which is the best algorithm, from among the six shown here, for each of the two kinds of activity? And, is the same algorithm the best in both cases?

For both issues, we have performed a suitable statistical analysis. Showing the whole set of related tables and findings would result in a too-high number of tables, which would be beyond the limit allowed by the journal. Hence, we show here a summary about our analysis. Interested readers may find in the below-mentioned papers a thorough description of the complete statistical analysis procedures followed here.

For the first issue, the Wilcoxon signed-rank test (Derrac et al., 2011) has been used. The choice of the Wilcoxon signed-rank test comes from the fact that here we wish to deal with repeated measurements over a same set of subjects, hence this test is well-suited. The most important reason here to prefer Wilcoxon to the *t*-test is that it is known that, whenever the sample sizes are small, say less than 30, the results of *t*-test can become little reliable. In this paper, we have small sets of samples, namely 15 subjects for each class and each test, so this is exactly the case. Moreover, unlike the *t*-test, for Wilcoxon there is no need to assume a normal distribution, and for it the outliers are of lower impact on the results than they are in t-test.

The article "The Effects of Physical Exercise on Cognition: How Heart Rate Variability Can Predict Cognitive Performances" was retracted in 2021. Reasons: results that could not be reproduced; errors in the methods.

The results of this test are reported in Table 6 and have shown that both kinds of physical activity are useful to improve cognitive performance. Namely, the aerobic activity of Group 1 (effort) has turned out to be statistically helpful for both tests related to planning, whereas the effort activity of subjects in Group 2 (aerobic) has proven statistically useful for all the three tests related to concentration. Finally, when all the subjects in both groups are considered together, all the three tests linked to concentration provide statistically superior results at the end of the study than they did at the beginning.

**Table 6:** Statistics of the Wilcoxon test for Group 1 (left), Group 2 (middle), and the two groups joined (right).

	**Group 1**			**Group 2**			**Group 1 & 2**		

	**w **%****	***w*_c_ %**		**w **%****	***w*_c_ %**		**w **%****	***w*_c_ %**	
Digit span	9	2	R	27	10	R	63.5	35	R
Monkey ladder	21.5	8	R	17.5	5	R	73.5	41	R
Paired association	17	10	R	3	3	NR	34	41	NR
Spatial span	20	8	R	20	10	R	87	53	R
Double trouble	0	17	NR	0	13	NR	0	83	NR
Gram. reasoning	24.5	13	R	24	17	R	94.5	83	R
Odd one out	34	13	R	25	10	R	104.5	67	R
Features match	15	17	NR	20	17	R	67.5	91	NR
Interlocking polygons	18.5	17	R	15	17	NR	63.5	91	NR
Spatial rotation	9	17	NR	7	17	NR	32	91	NR
Token search	36.5	17	R	22.5	8	R	111.5	67	R
Spatial planning	0	17	NR	0	13	NR	0	83	NR

For the second issue, instead, as we have reported the results of six different algorithms over a total of 12 tests, the use of non-parametrical statistical analysis is needed. By following (Demsar, 2006; Derrac et al., 2011), we have used Quade test, that takes account for the fact that not all the problems are equally difficult, or that the results obtained by the algorithms over them show larger differences, as it is the case here for the 12 cognitive tests. We have considered all the three quality indicators and all the subjects involved in this trial, and we have performed both the Quade statistical test and the related *post-hoc* procedures. The results over Group 1 (effort), shown in Tables 7, 8, reveal that Simple Linear is statistically better than the other five algorithms, followed by REPTree.

**Table 7:** The results of the Quade test for the three indicators for the subjects in Group 1.

	**Simple linear**	**REPTree**	**Additive**	**SVM**	**IBk**	**MLP**
Score	2.098	2.955	3.353	3.800	4.048	4.746
	**Statistic**: 11.598		***p*****-value**: 0.000			

The article "The Effects of Physical Exercise on Cognition: How Heart Rate Variability Can Predict Cognitive Performances" was retracted in 2021. Reasons: results that could not be reproduced; errors in the methods.

**Table 8:** *Post-hoc* procedure for Quade test over Group 1 subjects.

**Algorithm**	**p**	**z**	**Bonf**.	**Holm**	**Holl**.	**Rom**	**Finner**	**Li**
MLP	0.001	3.312	0.001	0.010	0.010	0.011	0.010	0.038
IBk	0.015	2.439	0.015	0.013	0.013	0.013	0.020	0.038
SVM	0.033	2.129	0.033	0.017	0.017	0.017	0.030	0.038
Additive	0.116	1.570	0.116	0.025	0.025	0.025	0.040	0.038
REPTree	0.284	1.072	0.284	0.050	0.050	0.050	0.050	0.050
Th			0.010	0.013	0.013	0.011	0.030	0.038

In the last row of Table 7, the value of the test statistic is also shown. This is a parameter specific to the particular statistical test executed. For the Quade test used in this paper, the test statistic is distributed according to an F-distribution with two degrees of freedom given by (number of algorithms - 1), and by (number of problems - 1) * (number of algorithms - 1), respectively. In this case, we have six algorithms and 12 problems (the 12 cognitive tests), so their values are equal to 5 and 175.

In the same row of the table, the corresponding *p*-value is shown. It represents the smallest level of significance that results in the rejection of the null hypothesis. This latter is a statement of no difference among the tested algorithms. Such a *p*-value is computed through the statistics of the test considered: low values strongly suggest the existence of significant differences among the algorithms considered.

As concerns Table 8, instead, the row at its bottom reports for each *post-hoc* procedure the threshold value Th. This is important because the procedure under account rejects those equivalence hypotheses characterized by an adjusted *p*-value lower than or equal to Th. Moreover, p represents the unadjusted *p*-value for the algorithm under account, as contrasted to the adjusted *p*-values resulting from the various *post-hoc* procedures used. Also, the variable z is the test statistic for this comparison, and its definition can be found in Derrac et al. (2011).

Over Group 2 (aerobic), instead, the results reported in Tables 9, 10 reveal that SVM turns out to be statistically better, REPTree being the runner up.

**Table 9:** The results of the Quade test for the three indicators for the subjects in Group 2.

	**SVM**	**REPTree**	**Simple linear**	**IBk**	**MLP**	**Additive**
Score	2.809	3.315	3.350	3.435	3.995	4.096
	**Statistic**: 4.533	***p*****-value**: 0.001				

**Table 10:** *Post-hoc* procedure for Quade test over Group 2 subjects.

**Algorithm**	**p**	**z**	**Bonf**.	**Holm**	**Holl**.	**Rom**	**Finner**	**Li**
Additive	0.108	1.609	0.108	0.010	0.010	0.011	0.010	0.025
MLP	0.138	1.483	0.138	0.013	0.013	0.013	0.020	0.025
IBk	0.434	0.782	0.434	0.017	0.017	0.017	0.030	0.025
Simp.Lin.	0.499	0.676	0.499	0.025	0.025	0.025	0.040	0.025
REPTree	0.527	0.632	0.527	0.050	0.050	0.050	0.050	0.050
Th			0.010	0.010	0.010	0.0	0.010	0.025

Given that we have obtained different conclusions when working with the two groups separately, the question arises about which the best algorithm is when all the subjects in the two groups are considered at the same time. Based on the results of the Quade statistical test shown in Tables 11, 12, the best-performing algorithm is, in this case, Simple Linear, REPTree being the runner-up.

The article "The Effects of Physical Exercise on Cognition: How Heart Rate Variability Can Predict Cognitive Performances" was retracted in 2021. Reasons: results that could not be reproduced; errors in the methods.

**Table 11:** The results of the Quade test for the three indicators for all the subjects.

	**Simple linear**	**REPTree**	**SVM**	**Additive**	**IBk**	**MLP**
Score	2.747	3.121	3.325	3.696	3.722	4.388
	**Statistic**: 11.034		***p*****-value**: 0.000			

**Table 12:** *Post-hoc* procedure for Quade test over all the subjects in Groups 1 and 2.

**Algorithm**	**p**	**z**	**Bonf**.	**Holm**	**Holl**.	**Rom**	**Finner**	**Li**
MLP	0.004	2.892	0.004	0.010	0.010	0.011	0.010	0.026
IBk	0.086	1.717	0.086	0.013	0.013	0.013	0.020	0.026
Additive	0.094	1.673	0.094	0.017	0.017	0.017	0.030	0.026
SVM	0.308	1.019	0.308	0.025	0.025	0.025	0.040	0.026
REPTree	0.510	0.659	0.510	0.050	0.050	0.050	0.050	0.050
Th			0.010	0.013	0.013	0.011	0.020	0.026

Actually, we have performed a much wider statistical analysis than reported here. In fact, for each indicator, and for each group, we have also considered three different statistical tests, i.e., Friedman, Aligned Friedman, and Quade (Derrac et al., 2011). Unfortunately, the paper would become too lengthy and would contain too many tables if we showed all of them here. In the following, we report a short summary of the results obtained in this way:

- Pearson for Group 1: for all the three statistical tests the best-performing algorithm turns out to be the SimpleLinear;
- Pearson for Group 2: all the three statistical tests conclude that the best-performing algorithm is IBk;
- MAE for Group 1: there are two algorithms that are statistically better, namely REPTree and SimpleLinear;
- MAE for Group 2: all the three statistical tests conclude that the best-performing algorithm is REPTree;
- RMSE for Group 1: SimpleLinear is statistically better for all the three statistical tests;
- RMSE for Group 2: all the three statistical tests conclude that the best-performing algorithm is REPTree.

## 4. Discussion

The importance of exercise to our overall well-being is well-documented in the scientific literature. It is recommended in the prevention and management of various medical conditions, including cardiovascular disease, metabolic syndrome, osteoporosis, and so on. Additionally, the benefits of exercise extend beyond physiological changes. Exercise also benefits mental health, having been shown to improve self-esteem and self-confidence and to reduce symptoms of depression.

The article "The Effects of Physical Exercise on Cognition: How Heart Rate Variability Can Predict Cognitive Performances" was retracted in 2021. Reasons: results that could not be reproduced; errors in the methods.

However, an often-overlooked aspect of exercise is the effect it has on cognition and the brain. Additionally, as far as reported in the literature, none of the published studies gives the possibility to predict the cognitive performance of the subjects. This possibility is what we investigate in this paper, and represents its novelty.

We have investigated the impact of physical activity on the cognitive performances measured by using a number of different cognitive tests taken from CBS. To do this, we have chosen to use the HRV, because the dynamic autonomic responses during exercise can be measured by analyzing the ECG signal, i.e., the HRV. In particular, we were interested in knowing whether HRV and variations in HRV parameters are associated with changes in the cognitive domain, that is, how the physical activity, measured by the variation in HRV, impacts on cognitive activities such as reasoning, work memory, and verbal skills.

We have performed the first analysis to determine whether the different exercise regimes (aerobic vs. effort exercise) had different effects on cognition. It has demonstrated that in most CBS tests there is an improvement, or at least a confirmation, of the subject's cognitive ability, both for effort workout (group 1) and for aerobic one (group 2). In particular, reasoning, concentration, and planning tests seem to undergo important positive changes due to physical exercise.

Secondly, a prediction analysis has been made in order to understand if, by monitoring the HRV during the exercise, it is possible to predict the cognitive performance, i.e., the CBS tests results. The regression analysis has demonstrated that this is possible to some extent, in terms of ρ, MAE, and RMSE. The results show that the best regression algorithm able to predict the cognitive performance by using the HRV is Simple Linear, or, subordinately, REPTre. Going into details, the best regression quality, in terms of ρ, MAE and RMSE, has been reached by a simple algorithm.

Summarizing, this study had numerous strengths, including the use of a large cognitive test battery, which allowed us to examine the effects of exercise on a range of cognitive functions. We compared two distinct exercise regimes, one of which focused on resistance exercise. The effects of long-term resistance exercise regimes have not been studied in healthy adults, and thus these results are novel.

The article "The Effects of Physical Exercise on Cognition: How Heart Rate Variability Can Predict Cognitive Performances" was retracted in 2021. Reasons: results that could not be reproduced; errors in the methods.

Additionally, as mentioned previously, no other studies have investigated the possibility of predicting cognitive abilities through a simple mathematical relationship expressed by Simple Linear. Our study suggests the possibility of using this model in a real-time mobile application that, monitoring HRV during exercise, could predict cognitive performance. If needed, this application could also suggest the subject to modify the physical training in order to improve the predicted cognitive performance. This app could be useful within cognitive rehabilitation, where only cognitive digital games are currently employed. In this way, to these latter an app-monitored personalized physical activity could be associated with maximizing cognitive improvements. Moreover, this app could also be applied to support active aging, so as to contribute to avoiding, or at least to slowing down, the onset of pathologies as, e.g., dementia, cognitive impairment, cognitive decline, and so on.

Despite these strengths, this study had limitations that should be addressed in the future. Among them, one is that no additional information, as for example the participant's diet, which is recognized in the literature as impacting mental health (Loughrey et al., 2017), was taken into consideration.

Additionally, the design of the study allowed us to examine the associations between cognition improvements and physical activity, but it did not allow us to establish the temporality of the observed relationships. As a consequence, we do not know if the effects of physical activity on cognition are short-term or last longer.

Finally, unfortunately, there is no guarantee about the applicability of our results, based on a sample of young and middle-aged adults, to older individuals. However, the results presented here are to be considered preliminary and could be used as a starting point for a new and more numerous pilot study. In fact, we plan to create a wider data set by enrolling more subjects representative of the population, and to make it available to the scientific community. This would allow us to create a freely available database on this specific problem.

## Data Availability Statement

The datasets used and/or analysed during the current study are available from the corresponding author on reasonable request.

## Ethics Statement

The studies involving human participants were reviewed and approved by CNR Ethics Committee. The patients/participants provided their written informed consent to participate in this study.

## Author Contributions

All authors contributed to the conception and the design of this study. Material preparation and data collection were performed by GS. Instead, the analysis was carried out by GS and ID. The first draft of the manuscript was written by GS and ID. All authors commented on the previous versions of this manuscript and read and approved the final manuscript.

The article "The Effects of Physical Exercise on Cognition: How Heart Rate Variability Can Predict Cognitive Performances" was retracted in 2021. Reasons: results that could not be reproduced; errors in the methods.

## Conflict of Interest

The authors declare that the research was conducted in the absence of any commercial or financial relationships that could be construed as a potential conflict of interest.

## Footnotes

^1^www.cambridgebrainsciences.com

^2^www.cambridgebrainsciences.com

^3^www.cambridgebrainsciences.com
